# Research on Transboundary Regulation of Plant-Derived Exogenous MiRNA Based on Biological Big Data

**DOI:** 10.1155/2021/6656763

**Published:** 2021-01-31

**Authors:** Zhi Li, Xu Wei, Shuyi Li, Jiashi Zhao, Xiang Li, Liwan Zhu

**Affiliations:** ^1^School of Computer Science and Technology, Changchun University of Science and Technology, Changchun 130022, China; ^2^College of Computer Science and Technology, Jilin University, Changchun 130012, China; ^3^School of Foreign Languages, Harbin Institute of Technology, Harbin 150001, China

## Abstract

In recent years, researchers have discovered plant miRNA (plant xenomiR) in mammalian samples, but it is unclear whether it exists stably and participates in regulation. In this paper, a cross-border regulation model of plant miRNAs based on biological big data is constructed to study the possible cross-border regulation of plant miRNAs. Firstly, a variety of human edible plants were selected, and based on the miRNA data detected in human experimental studies, screening was performed to obtain the plant xenomiR that may stably exist in the human body. Then, we use plant and animal target gene prediction methods to obtain the mRNAs of animals and plants that may be regulated, respectively. Finally, we use GO (Gene Ontology) and the Multiple Dimensional Scaling (MDS) algorithm to analyze the biological processes regulated by plants and animals. We obtain the relationship between different biological processes and explore the regulatory commonality and individuality of plant xenomiR in plants and humans. Studies have shown that the development and metabolic functions of the human body are affected by daily eating habits. Soybeans, corn, and rice can not only affect the daily development and metabolism of the human body but also regulate biological processes such as protein modification and mitosis. This conclusion explains the reasons for the different physiological functions of the human body. This research is an important meaning for the design of small RNA drugs in Chinese herbal medicine and the treatment of human nutritional diseases.

## 1. Introduction

MicroRNA (miRNA) is a type of noncoding single-stranded small RNA with a size of 21–23 nucleotides. It binds to mRNA through the base complementation rule, degrades mRNA, inhibits mRNA translation, and ultimately regulates gene expression [1]. It plays a role in all aspects of the life cycle of biological cells. With the development of genome sequencing technology and the emergence of miRNA verification methods based on high-throughput biological big data, researchers have discovered more miRNAs and studied them in depth. The expression regulation function of miRNA has become a research hotspot in this field [2].

Studies have shown that miRNAs can not only function in their own body but also perform cross-border regulation. As an exogenous biological activity unit, it can affect the expression of heterologous mRNA through base complementation.

In the process of studying the regulatory functions of miRNAs, plant miRNAs were found in mammalian samples [3–8]. Researchers infer that these plant miRNAs enter the animal's body through food. Researchers call these exogenous miRNAs of plant origin (plant xenomiR).

Although there are many studies on plant xenomiR transboundary regulation, they are all based on a single plant miRNA. However, studies have found that not all plant miRNAs can enter the human body. The human body specifically absorbs plant miRNA. Therefore, it is meaningful to select plant miRNAs that exist in animals for subsequent analysis. The determination of plant xenomiR is the key to this research [9–11].

In this article, on the basis of plant xenomiR transboundary regulation, a research model of plant xenomiR transboundary regulation based on biological big data is proposed and constructed. The possible regulatory functions of plant XenomiR in animals and plants were studied, respectively, and the Multiple Dimensional Scaling (MDS) algorithm was used to analyze the regulatory functions of different species, to study the cross-species regulation mechanism of XenomiR on different kinds of edible plants. Not only the regulation effect of plant xenomiR on the plant body but also its regulation effect on the human body can be obtained. Explore these plant xenomiR regulatory characteristics. This model can be applied to the research of cross-species regulation mechanism, Chinese herbal medicine efficacy, nutrition, and other fields.

## 2. Materials and Methods

### 2.1. Technical Route

In this paper, a research model of plant xenomiR transboundary regulation based on biological big data is constructed. Firstly, select the miRNA data of various human edible plants, and use the miRNA data detected in the human body obtained by the second-generation sequencing technology to perform data screening to obtain the plant xenomiR data present in human samples. Then, using plant and animal target gene prediction methods, the plant and animal mRNA that may be regulated are obtained, respectively. Finally, perform functional analysis of mRNA, use GO enrichment analysis and the Multiple Dimensional Scaling (MDS) algorithm to analyze its biological processes in plants and animals from the same perspective, and obtain the relationship between different biological processes. Look for the regulatory commonalities and individualities of plant miRNAs that coexist in plants and humans.

The technical route is shown in Figure 1.

1. Data acquisition: choose a variety of plants that are edible by humans. Obtain human miRNA second-generation sequencing data, miRNA sequence data, and mRNA data of related plants from professional public databases and literature data. Search for data related to plant miRNA in human miRNA second-generation sequencing data.
2. Target gene prediction: use the target gene prediction algorithm for xenomiR mRNA comparison and statistical screening to obtain the target gene data of plant xenomiR in plants and humans.
3. Core node screening: use the LeaderRank algorithm to calculate the score of each node and find the core node of the network.
4. Core network construction and function enrichment analysis: build a biological regulatory network through core nodes and combine it with function enrichment analysis to study the similarities and differences between these miRNAs participating in the biological processes of plants and humans.
5. GO analysis: analyze the similarities and differences of the data in different comparison groups, and analyze the GO semantic relationship of these data by using the MDS algorithm. Explore the commonalities and individual differences of its function of gene regulation.

### 2.2. Data Acquisition and Preprocessing

Data needed for study: miRNA and mRNA of edible plants (soybean, rice, and corn), sequencing data based on high-throughput human miRNA, human mRNA data, gene annotation files of edible plants and humans.

The miRNA data of plant crops comes from the miRBase database (http://www.mirbase.org/); the database version is 22.1 (October 2018). The study is to explore the role of plant miRNAs obtained by humans through food. Therefore, the necessary conditions for selecting crops for research are as follows: crops that are often eaten by humans in daily life and related data are perfect for subsequent analysis. After screening, the final eligible crops are as follows: soybeans, rice, and corn.

Related information is shown in Table 1.

The research needs to obtain plant miRNA data found in human samples. Qi Zhao and others in our laboratory analyzed 388 human small RNA sequencing data and detected a total of 484 plant miRNAs, including 166 unique miRNA sequences [12].

The relevant plant mRNA data were downloaded from NCBI (https://www.ncbi.nlm.nih.gov/), and the human mRNA data were downloaded from GENCODE (https://ucscgenomics.soe.ucsc.edu/gencode/). The relevant data statistics are shown in Table 2.

Compare the obtained miRNA data of soybean, rice, and corn with the 166 plant miRNA data found in human samples to obtain the source of plant xenomiR. The statistical results are shown in Table 3.

### 2.3. Target Gene Prediction

Find the target genes of plants and humans corresponding to the target of the corresponding plant xenomiR.

In this paper, the tapir algorithm based on RNAHybrid was used to predict the target gene [13, 14]. The Tapir algorithm can set its own parameters to make the results more accurate. The Tapir algorithm is specially designed for plant miRNAs and has a good predictive effect on plant miRNA target genes. The screening criteria used are as follows: exact match of seed region; remove the results with more than 3 bases of mismatches; set the MFE (minimum free energy) threshold of the result to −25; and set the *p*_*value* threshold to 0.05. When the above conditions are met, it is deemed to meet the standards.

The prediction process used in this paper is shown in Figure 2.

The relevant statistical results are shown in Table 4.

Since three edible plants were selected in this article, all experimental results in this article are divided into six groups.

### 2.4. Core Node Screening

The currently acquired data contains a large number of independent nodes or nodes that are not closely related to other network nodes. This information makes the biological pathways unobvious and fails to reflect the core of the network, making it difficult to understand the regulatory network. Therefore, it is necessary to find the core node after filtering the nodes.

The LeaderRank algorithm is used to score and rank the nodes required by the biological regulatory network. It adds the background node *b* based on the PageRank algorithm and connects it with other nodes to form a strong connection graph. The degree of each node is greater than 0, to avoid the existence of isolated nodes, so that the results can converge faster [15, 16].

Set the LeaderRank score of node *b* as *S*_*b*_=0 and the scores of other *n* nodes as *S*_*i*_=1, through the iterative formula:

(1) $$\begin{array}{c} S_{i}\left(t\right)=\overset{n+1}{\underset{j=1}{\sum }}\frac{a_{ji}}{O_{j}}S_{j}\left(t-1\right). \end{array}$$

After the element value gradually converges, we use *t*_*c*_ to represent the number of convergence and then obtain the score of each node:

(2) $$\begin{array}{c} S_{i}=S_{i}\left(t_{c}\right)+\frac{S_{b}\left(t_{c}\right)}{n}. \end{array}$$

After using the above method to operate, the changes in the number of nodes before and after are shown in Table 5.

### 2.5. GO Analysis Based on Multiple Dimensional Scaling Algorithm

By performing functional enrichment analysis on multiple sets of data, information such as the contained biological processes can be obtained. However, usually due to the diversity of results, it is difficult to dig out meaningful biological information from a large amount of information.

The dimensionality reduction processing of the data through the MDS algorithm can ensure that the distance between the data samples after dimensionality reduction does not change compared with that before dimensionality reduction, which is very helpful for GO semantic analysis [17].

In the MDS algorithm, assuming that there are *m* samples in the data, their sample space is

(3) $$\begin{array}{c} T=\left\{x_{1},\right.\left.x_{2},x_{3},x_{4},\ldots ,x_{m},\right\}\;x_{i}\in R^{d}. \end{array}$$

Assuming that the matrix *D* is the distance between samples and D ∈ *R*^*m*×m^, the distance between sample *x*_*i*_ and sample *x*_*j*_ is the element *d*_*ij*_ in D. The sample in the new space can be expressed as

(4) $$\begin{array}{c} Z\in R^{d^{\prime }\times m},\\ d^{\prime }\leq d. \end{array}$$

The Euclidean distance between the new and old data in the two spaces is the same as

(5) $$\begin{array}{c} Z_{i}-Z_{j}=d_{ij}. \end{array}$$

Let the inner product matrix of the sample after dimensionality reduction be

(6) $$\begin{array}{c} B=Z^{T}Z\in R^{m\times m}. \end{array}$$

And *b*_*ij*_=*Z*_*i*_^*T*^*Z*_*j*_; then,

(7) $$\begin{array}{c} d_{ij}^{2}=Z_{i}{}^{2}+Z_{j}{}^{2}-2Z_{i}^{T}Z_{j}=b_{ii}+b_{jj}-2b_{ij}. \end{array}$$

When the sample *Z* after dimensionality reduction is centered ∑_*i*=1_^*m*^*Z*_*i*_=0, the sum of the rows and columns of matrix B is 0; that is,

(8) $$\begin{array}{c} \overset{m}{\underset{i=1}{\sum }}b_{ij}=\overset{m}{\underset{j=1}{\sum }}b_{ij}=0. \end{array}$$

When using *tr* () to represent the matrix,

(9) $$\begin{array}{c} trB=\overset{m}{\underset{j=1}{\sum }}Z_{i}^{2}. \end{array}$$

Available:

(10) $$\begin{array}{c} \overset{m}{\underset{i=1}{\sum }}d_{ij}^{2}=tr\left(B\right)+mb_{jj}, \end{array}$$

(11) $$\begin{array}{c} \overset{m}{\underset{j=1}{\sum }}d_{ij}^{2}=tr\left(B\right)+mb_{ii}, \end{array}$$

(12) $$\begin{array}{c} \overset{m}{\underset{i=1}{\sum }}\overset{m}{\underset{j=1}{\sum }}d_{ij}^{2}=2mtr\left(B\right). \end{array}$$

Make

(13) $$\begin{array}{c} d_{i.}^{2}=\frac{1}{m}\overset{m}{\underset{j=1}{\sum }}d_{ij}^{2}, \end{array}$$

(14) $$\begin{array}{c} d_{..}^{2}=\frac{1}{m^{2}}\overset{m}{\underset{i=1}{\sum }}\overset{m}{\underset{j=1}{\sum }}d_{ij}^{2}. \end{array}$$

In summary,

(15) $$\begin{array}{c} b_{ij}=-\frac{1}{2}\left(d_{ij}^{2}-d_{i.}^{2}-d_{.j}^{2}+d_{..}^{2}\right). \end{array}$$

In this algorithm, *D* is kept unchanged, that is, the distance between samples is unchanged, and so the inner product matrix B can be calculated by D. At the same time, because B is a symmetric matrix, it can be feature decomposition, and we can get

(16) $$\begin{array}{c} B=V\Delta V_{T}, \end{array}$$

where ∧ is the diagonal matrix, which is composed of eigenvalues, and *V* is the corresponding eigenvector matrix.

Assuming that there are *d*_*∗*_ nonzero eigenvalues, they can form a diagonal matrixΛ_*∗*_. Assuming Λ_*∗*_ is the corresponding eigenvector matrix, the sample in the new space represents *Z*:

(17) $$\begin{array}{c} Z=\Lambda_{*}^{1/2}V_{*}^{T}\in R^{d^{*}\times m}. \end{array}$$

## 3. Results and Discussion

### 3.1. Functional Enrichment Analysis of Plant-Plant Group

For the plant's own regulation mode, we select the data with *p*_value ≤ 0.05 for analysis, take  log_10_ *p*_value, and sort them from large to small, combined with the number of genes in the relevant biological process.

The statistical results of soybean-soybean biological process information are shown in Figure 3.

The statistical results of the soybean protein interaction network are shown in Figure 4.

The statistical results of rice-rice biological process information are shown in Figure 5.

The statistical results of the rice-protein interaction network are shown in Figure 6.

The statistical results of corn-corn biological process information are shown in Figure 7.

The statistical results of the corn protein interaction network are shown in Figure 8.

### 3.2. Functional Enrichment Analysis of Plant-Human Group

In the experiment of plant and colleagues, the data *p*_value ≤ 0.05 are also selected for analysis.

The statistical results of soybean-human biological process information are shown in Figure 9.

The statistical results of the soybean-human protein interaction network are shown in Figure 10.

According to its biological process information, rice has a particularly obvious regulation in human development. The protein interaction network for nervous system development is shown in Figure 11.

The statistical results of rice-human biological process information are shown in Figure 11.

The statistical results of rice-human-protein interaction network are shown in Figure 12.

The statistical results of corn-human biological process information are shown in Figure 13.

The statistical results of corn-human-protein interaction network are shown in Figure 14.

### 3.3. Biological Process and GO Semantic Analysis

In the GO semantic analysis graph, color is used to represent the change of log_10_ *p*_*value*, the larger the value, the warmer the color, and the radius is used to represent the value of log *size*.

#### 3.3.1. Soybean

Soybean miRNAs play different regulatory roles in plants and humans, and their regulatory roles in humans are quite different.

Soybean miRAN plays a regulatory role in soybean that is mostly related to plant development, such as leaf development, integument development, another development, and positive developmental regulation (see Figure 15).

The regulatory role of soybean miRNA in the human body is related to cell protein modification process, cell response to external stimuli, cell protein metabolism process, protein ubiquitination, regulation of mitotic cell cycle, and so forth. There is no obvious correlation between various biological processes (see Figure 16).

#### 3.3.2. Rice

Rice miRNAs regulate the biological metabolism and development of rice itself, as well as humans. At the same time, it can also regulate the response of cells to external stimuli, cell processes, and cell communication.

Most of the regulatory effects of rice miRNA are related to metabolism and development. Metabolism includes the metabolic process of cellular aromatic compounds, the metabolic process of organic cyclic compounds, the cellular metabolic process, the cellular macromolecular metabolic process, and the organic matter metabolic processes. Development-related includes multicellular organism development, flower development, postembryonic development, system development, organ development, reproductive system development, postembryonic organ development, and tissue development (see Figure 17)

Most of the regulatory effects of rice miRNA in the human body are also related to metabolism and development. Metabolism includes organic matter metabolism, primary metabolism, cellular macromolecular metabolism, cell metabolism, nitrogen compound metabolism, and phosphorus metabolism process. Development-related includes nervous system development, neuron production, cell differentiation, brain development and ventricular system development, and lateral ventricle development. At the same time, it can also regulate the response of cells to stimuli and regulate cell processes, cell-to-cell communication, and cell division cycles (see Figure 18).

#### 3.3.3. Corn

Maize miRNAs can regulate metabolism in both plants and humans, and they can also regulate biological processes.

Most of the regulatory effects of maize miRNA in maize are related to metabolism and transcription and translation, such as lignin catabolism, phenyl propane catabolism, cellular aromatic compound metabolism, phenyl propane metabolism, and organic cyclic compound metabolism. Transcription and translation-related include nucleic acid template transcription, biosynthetic process, nucleic acid template transcription, regulation of gene expression in biosynthesis process, regulation of nucleic acid template transcription, and regulation of RNA biosynthesis process (see Figure 19).

The miRNA of corn can regulate the response to stimuli in the human body, such as cell response to endogenous stimuli, cell response to peptide hormone stimulation, cell response to growth factor stimulation, cell response to organic matter, and cell response reaction to chemical stimuli. It can regulate metabolism, such as cell protein metabolism process, positive regulation of phosphoric acid metabolism process, and organic nitrogen compound metabolism process. It can regulate cell functions, such as regulation of multicellular tissue processes and regulation of cytokine production (see Figure 20).

## 4. Conclusions

By research, it is found that, in terms of plant xenomiR's, common regulation of humans, soybean, rice, and corn all, contain miRNAs that can regulate the daily development and metabolism of the human body. These miRNAs can also regulate other biological processes, such as response to external stimuli (GO: 0051716), protein modification (GO: 0006464), and mitotic cell cycle (GO: 0007346).

In terms of personality regulation, soybean can regulate the process of protein ubiquitination (GO: 0016567), which plays an important role in protein metabolism and degradation and also participates in cell proliferation and differentiation, repairing damage, and immune inflammation. Rice is particularly effective in regulating human development, such as nervous system development (GO: 0007399), brain development (GO: 0007420), and ventricular system development (GO: 0021591). Corn has a regulatory effect on protein phosphorylation (GO: 0001932), which can regulate the activity and function of the protein, which is the most common and important regulatory mechanism.

This shows that when humans eat plants, the development and metabolic functions of the human body will be affected accordingly, and various physiological functions will also change. And due to different eating habits, the possible adjustments will also be different.

This conclusion explains the different effects of daily eating habits on the physiological functions of the human body, which is consistent with the experimental research results of Sanchta [18]. Plant xenomiR can play a role in the human body, and edible plant xenomiR can be used as a nutritional supplement, which can bring beneficial effects to human health.

## Figures and Tables

**Figure 1:** Research model of plant xenomiR transboundary regulation based on biological big data.

**Figure 2:** Plant xenomiR target gene prediction process.

**Figure 3:** Soybean-soybean biological process information statistics map (total of 33 items).

**Figure 4:** Soybean protein interaction network.

**Figure 5:** Rice-Rice biological process information statistics map (total of 59 items).

**Figure 6:** Rice-protein interaction network (metabolism-related).

**Figure 7:** Corn-corn biological process information statistics map (total of 37 entries).

**Figure 8:** Corn protein interaction network.

**Figure 9:** Soybean-human biological process information statistics map (total of 7 entries).

**Figure 10:** Soybean-human protein interaction network (related to protein ubiquitination).

**Figure 11:** Rice-human biological process information statistics map (total of 90 entries showing only partial information).

**Figure 12:** Rice-human-protein interaction network (related to nervous system development).

**Figure 13:** Corn-human biological process information statistics map (total of 86 entries showing only partial information).

**Figure 14:** Corn-human-protein interaction network.

**Figure 15:** Soybean-soybean GO semantic analysis diagram.

**Figure 16:** Semantic analysis diagram of soybean-human GO.

**Figure 17:** Semantic analyses of rice GO.

**Figure 18:** Semantic analysis diagram of rice-human GO.

**Figure 19:** Semantic analysis diagram of corn-maize GO.

**Figure 20:** Semantic analysis diagram of corn-human GO.

**Table 1:** Plant information table.

Name	Scientific name	Quantity
Soybeans	*Glycine max* (Linn.) Merr.	756
Rice	*Oryza sativa japonica* group	738
corn	*Zea mays* Linn.	325

**Table 2:** Plant, crop, and human mRNA data.

Species name	Soybean	Rice	Corn	Human
Quantity	71149	42474	56152	206694

**Table 3:** Statistics of plant xenomiR.

Plant name	Soybean	Rice	Corn
Quantity	42	46	29
Percentage	5.56%	6.23%	8.92%

**Table 4:** Statistics of target gene prediction results.

	Soybean-soybean	Rice-rice	Corn-corn	Soybean-person	Rice-person	Corn-person
Target	1119	767	443	1419	2409	1343
GeneID	380	396	214	378	632	358

**Table 5:** Statistics of the number of nodes before and after screening.

	Soybean-soybean	Rice-rice	Corn-corn	Soybean-person	Rice-person	Corn-person
Before screening	380	396	214	378	632	358
After screening	156	129	54	260	231	43

## Data Availability

All personnel can access the data that include plant miRNA and mRNA information and related processing procedures. The data download address is https://pan.baidu.com/s/1YlOzS4LsWEmQNuTln7yemA with code ‘5b2e'.
